# A negative feedback loop between long noncoding RNA NBAT1 and Sox9 inhibits the malignant progression of gastric cancer cells

This article has been retracted.

**DOI:** 10.1042/BSR20180882

**Published:** 2018-11-16

**Authors:** Jijun Yan, Wenwei Huang, Xiufang Huang, Wencai Xiang, Chao Ye, Juntao Liu

**Affiliations:** Department of General Surgery, Hanchuan People’s Hospital, Hubei Province, China

**Keywords:** angiogenesis, feedback, NBAT1, Sox9

## Abstract

Long noncoding RNAs (lncRNAs) play critical roles in carcinogenesis and progression, and act as important gene expression modulators. Recent evidence indicates that lncRNA neuroblastoma associated transcript 1 (NBAT1) functions as a tumor suppressor in some types of human cancers. However, its functional role in the development of gastric cancer (GC) remains unknown. The aim of this research was to investigate the clinical significance and biological functions of NBAT1 in GC. NBAT1 was found to be significantly down-regulated in GC tissue. Decreased NBAT1 expression was correlated with poor differentiation, higher tumor stage and lymph node metastasis, and poor prognosis. Functional assays showed that NBAT1 inhibited GC proliferation, migration, and invasion. NBAT1 also suppressed proliferation, migration, and capillary tube formation of human umbilical vein endothelial cells (HUVECs). Mechanistically, NBAT1 interacted with Sox9, and reduced its protein stability by promoting it from polyubiquitination and proteasome-dependent degradation. Moreover, we revealed that Sox9 could occupy the NBAT1 promoter to inactivate its transcription. The negative feedback loop of NBAT1 and Sox9 continuously enhanced the suppressive effects. In conclusion, these findings suggest that feedback regulation of NBAT1 and Sox9 served as a critical effector in GC progression.

## Introduction

Gastric cancer (GC) is one of the most prevalent malignant cancers and the second leading cause of cancer-associated deaths worldwide [1,2]. Due to nonspecific symptoms in the early stage, GC patients are always diagnosed in an advanced stage. Recently, despite the great advances in therapeutic approaches of GC, including surgery, chemotherapy, radiotherapy, and novel targetted therapy, the overall survival rates for these patients remain unsatisfactory [3]. Hence, great efforts should be obtained to reveal the key mechanisms underlying GC progression and provide novel promising therapeutic targets.

Growing evidence has highlighted that long noncoding RNAs (lncRNAs) play important roles in both physiological and pathological processes [4]. Growing evidence has highlighted that lncRNAs play important roles in both physiological and pathological processes. lncRNAs regulate gene expression through interacting with different molecules. For example, lncRNAs associate with DNA-binding proteins, such as transcription factors and chromatin-modifying complexes, and induce epigenetic alterations. lncRNAs function as molecular miRNAs sponge to modulate mRNA degradation and translation. Moreover, lncRNAs are involved in protein modification, such as phosphorylation and ubiquitination [5,6]. Deregulated expression of lncRNAs has been found during GC development and progression. For instance, lncRNA GALNT5 uaRNA is markedly up-regulated in GC relative to corresponding normal gastric tissues and correlated with the TNM stage and with lymph node metastasis. GALNT5 uaRNA facilitates the proliferation and migration of GC cells via binding with HSP90 [7]. Therefore, identifying crucial functional lncRNAs will be important for better revealing the underlying mechanism during GC pathogenesis.

A genome-wide association study identifies a susceptibility locus to clinically aggressive neuroblastoma at 6p22 [8]. Recently, lncRNA neuroblastoma associated transcript 1 (NBAT1), transcribed from the intron of chromosome 6p22, has been functionally characterized. NBAT1 functions as a tumor suppressor in several cancers, such as osteosarcoma, neuroblastoma, and breast cancer. NBAT1 inhibits cell proliferation, migration, and invasion through interaction with EZH2 and *miR-21* [9–12]. However, the functional significance of NBAT1 in GC progression remains unknown.

In the current research, we investigated the expression of NBAT1 in GC tissues and cells. NBAT1 was overexpressed and silenced in GC cells to determine the effect of NBAT1 in regulating GC cell proliferation, apoptosis, migration, and angiogenesis. Moreover, we found that NBAT1 exerted tumor-suppressive activity through degrading Sox9 protein. Our findings contributed to a better understanding of lncRNA functions in GC.

## Materials and methods

### Tissues’ collection and cell culture

GC tumoral and their corresponding adjacent nontumoral tissues were obtained from Hanchuan People’s Hospital between 2010 and 2016. All patients gave informed consent. The GC patients were diagnosed via histopathological detection. The present study was approved by the Research Ethics Committee of Hanchuan People’s Hospital. SGC7901, BGC-823, MGC803, MKN28, and AGS cell lines and a normal gastric epithelium cell line (GES-1) were purchased from the Cell Bank of the Chinese Academy of Sciences (Shanghai). Human umbilical vein endothelial cells (HUVECs) were also purchased from the Cell Bank of the Chinese Academy of Sciences (Shanghai). All cells were cultured in DMEM with 10% FBS (Invitrogen) at 37°C in 5% CO_2_.

### Cell proliferation assay

Cell proliferation was determined by CCK-8 and colony formation assays. For CCK-8 assay, 3 × 10^3^ cells per well were seeded in 96-well plates. At indicated time point, the cell proliferation was detected by the CCK-8 assay kit at 450 nm in a microplate absorbance reader (Bio-Rad). For colony formation assay, a total of 2 × 10^3^ cells per well were seeded in six-well plates and cultured. After 2 weeks of culture, cell clones were fixed and then stained with 0.5% Crystal Violet.

### Cell apoptosis

For cell apoptosis detection, GC cells were stained by Annexin V and propidium iodide (PI) using the Annexin V–FITC Apoptosis Detection kit (Dojindo), and the apoptosis was examined by FACS Calibur system (Beckman Coulter).

### Migration and invasion assay

The transwell assay was used to evaluate cell migration and invasion as manufacturer’s instruction. For migration assay, 1.0 × 10^5^ cells were seeded in serum-free medium in the top chamber, while the DMEM containing 10% FBS was placed in the lower chamber. For invasion assay, 2 × 10^5^ cells were seeded in serum-free medium in the top chamber coated with Matrigel, while the DMEM containing 10% FBS was placed in the lower chamber. After incubation for 12 h, cells remaining in the upper chamber were wiped off, and cells in the lower chamber were fixed with 4% paraformaldehyde and stained with Crystal Violet. Number of cells migrating or invading across membrane in ten random fields were counted.

### Transfection

Full-length NBAT1 or Sox9 were cloned into pcDNA3.1 plasmid. shRNA targetting NBAT1 was inserted into pLKO.1 plasmid. The target sequence of NBAT1 shRNA was shown as follows: CAGGCAGATACATCAGATA. Plasmid expressing NBAT1, Sox9, or NBAT1 shRNAs was transfected into GC cells by using the Lipofectamine 3000 kit (Invitrogen) according to the manufacturer’s instructions. After 48 h of transfection, cells were harvested for further detection, such as CCK-8 and apoptosis analysis.

### RNA extraction and quantitative real-time PCR

Total RNA was isolated using TRIzol reagent (Invitrogen) according to the standard protocols. Reverse transcription was performed by M-MLV reverse transcriptase (Invitrogen). The RNA expression levels were determined by using SYBR Green assays (TaKaRa) on ABI 7900HT Real-Time PCR System (Applied Biosystems, U.S.A.). The primer sequences were provided as follows: NBAT1, forward (5′-GAGAGACAAACAGGGTCAACTC-3′) and reverse (5′-CTGATGCCCAGAACCAAAGA-3′); Sox9, forward (5′-TCTGGAGACTTCTGAACGAGAG-3′) and reverse (5′-TCTGGAGACTTCTGAACGAGAG-3′); GAPDH, forward (5′-CCCTTCATTGACCTCAACTACA-3′) and reverse (5′-ATGACAAGCTTCCCGTTCTC-3′). GAPDH was used as the internal control. Comparative quantitation was determined using the 2^−ΔΔ*C*^_T_ method.

### RNA immunoprecipitation and RNA pull-down

RNA immunoprecipitation (RIP) and RNA pull-down assays were performed to examine the association between Sox9 and NBAT1 by using the Magna RIP™ RNA-Binding Protein Immunoprecipitation Kit (Millipore) and Magnetic RNA-Protein Pull-Down Kit (Thermo Fisher) according to the manufacturers’ protocols, respectively.

### Western blot

Protein samples were run on SDS/PAGE, and then transferred to PVDF membranes (Millipore). After blocking, the membranes were incubated with the primary antibodies against Sox9 (AB5535, Millipore), ubiquitin (3936, Cell Signaling Technology), and β-actin (3700, Cell Signaling Technology) overnight and then incubated with horseradish peroxidase–conjugated secondary antibody for 1 h at room temperature. The protein was measured with ECL substrate kit (Millipore).

### Luciferase reporter assay

The pGL3 luciferase reporter plasmid containing a 2-kb fragment (−1 to −2000 nts) of the NBAT1 promoter (pGL3-NBAT1) was constructed. Control and NBAT1 overexpressing AGS cells were transfected with pGL3 or pGL3-NBAT1 along with *Renilla* luciferase expressing plasmid using Lipofectamine 2000 (Invitrogen). Two days later, cells were lysed using 1× passive lysis buffer (#E194, Promega) and lysates were analyzed using the Dual-Luciferase Reporter Assay System (#E1960, Promega).

### Tube formation assay

Forty-eight well culture plates were precoated with 5  mg/ml Matrigel (BD Biosciences,) per well at 37 °C for 30 min for hardening. Confluent cells were suspended in tumor conditioned medium at the density of 1.5  ×  10^5^ cells/ml at 37 °C for 24  h. The resulting capillary-like structures were then photographed using Olympus DP71 immunofluorescence microscopy and were measured. Number of capillary-like structures in ten random fields were counted.

### *In vivo* ubiquitination assay

Endogenous Sox9 was immunoprecipited using the anti-Sox9 antibody (AB5535, Millipore) in denaturing conditions. The purified Sox9 protein was subjected to Western blot analysis and immunoblotted with anti-ubiquitin antibody (3936, Cell Signaling Technology).

### ChIP assay

ChIP assays were performed using the EZ Magna ChIP Kit (Millipore) as in its manual. Briefly, cells were cross-linked and then sonicated into DNA fragments. Anti-Sox9 antibody and negative control normal IgG were used for each immunoprecipitation. Immunoprecipitated and input DNAs were subjected to quantitative real-time PCR (qRT-PCR) analysis.

### Statistical analysis

Statistical analysis was performed using the SPSS software (version 11.0). Chi-square was used to analyze the correlation between NBAT1 expression and clinical features of GC patients. Student’s *t* test or one-way ANOVA was used for comparison amongst different groups. *P*<0.05 was considered significant.

## Results

### Down-regulation of NBAT1 is associated with poor prognosis of GC patients

We first investigated NBAT1 levels in a cohort of 78 paired GC tumoral and corresponding adjacent nontumoral tissues using qRT-PCR. As shown in Figure 1A, NBAT1 expression was significantly lower in the tumoral tissues. Next, we examined NBAT1 expression in GC cell lines (SGC7901, BGC-823, MGC803, MKN28, and AGS) and normal gastric epithelium cells GES-1 using qRT-PCR. NBAT1 was expressed at lower levels in major GC cells compared with the GES-1 cells (Figure 1B). Collectively, these results show that NBAT1 is down-regulated in GC tissues and cells.

**Figure 1:** Down-regulation of NBAT1 is associated with poor prognosis of GC patients (**A**) NBAT1 expression was determined in 78 paired GC tumoral and corresponding adjacent nontumoral tissues using qRT-PCR. (**B**) The NBAT1 expression in different cell lines. (**C**) The correlation between NBAT1 and prognosis of GC patients was analyzed by Kaplan–Meier survival analysis.

To investigate the association between NBAT1 expression and clinical characteristics, GC patients were divided into two groups: the low NBAT1 expression group (*n*=44, fold-change ≤2) and the high NBAT1 expression group (*n*=34, fold-change ≥2). As shown in Table 1, down-regulation of NBAT1 indicated poor differentiation, higher tumor stage and lymph node metastasis in GC patients. However, other factors showed no significant correlation. Then, a Kaplan–Meier survival analysis was performed to examine the correlation between NBAT1 expression and the prognosis of patients with GC. The results showed that patients with lower NBAT1 levels had shorter overall survival time than those with higher NBAT1 levels (Figure 1C). These findings suggest that NBAT1 may act as a tumor suppresser in the pathogenesis of GC.

**Table 1:** The correlation between NBAT1 expression and clinical parameter of GC patients

Clinical parameter	NBAT1 expression		*P*-value
	Low (*n*=44)	High (*n*=34)	
Age (years)			
>60	34	20	0.216
<60	10	14	
Gender			
Male	28	20	0.757
Female	16	14	
Tumor sizes			
>5 cm	24	16	0.737
<5 cm	20	18	
Tumor location			
Distal	36	26	0.691
Proximal	8	8	
Differentiation			
Well to moderate	14	20	0.017
Poor	30	14	
Lymph node metastasis			
Negative	8	20	0.008
Positive	36	14	
TNM stages			
I, II	6	16	0.021
III, IV	38	18	

### NBAT1 suppresses proliferation and induces apoptosis in GC cells

Next, we investigated the role of NBAT1 in GC progression. Given the endogenous NBAT1 expression, we overexpressed NBAT1 in BGC-823, silenced NBAT1 in AGS cells (Figure 2A,B). The CCK-8 assays showed that NBAT1 shRNAs significantly enhanced the proliferation of AGS cells, while NBAT1 overexpression decreased the proliferative capacity of BGC-823 cells (Figure 2C,D). Consistent with the results of CCK-8 assays, colony formation analysis demonstrated that NBAT1 knockdown increased clone formation of AGS cells, whereas NBAT1 overexpression dramatically suppressed the colony formation capacity of the BGC-823 cells (Figure 2E,F). We then performed flow cytometry analysis to determine whether NBAT1 is involved in regulating cell apoptosis. Deletion of NBAT1 significantly reduced the cell apoptotic rate of AGS cells, while up-regulation of NBAT1 increased BGC-823 cell apoptosis (Figure 2G,H). These results suggest that NBAT1 is involved in the growth of GC cells.

**Figure 2:** NBAT1 suppresses proliferation and induces apoptosis in GC cells (**A**) The validation of stably overexpressing NBAT1 in BGC-823 cells. (**B**) The validation of stably knocked down NBAT1 in AGS cells. (**C**) Proliferation assay of AGS cells with NBAT1 knockdown via CCK-8 detection. NC indicates negative control. shNBAT1 represents NBAT1 knockdown by shRNAs. (**D**) Proliferation assay of BGC-823 cells with NBAT1 overexpression via CCK-8 detection. CTR indicates the control group, and NBAT1 refers to NBAT1 overexpression. (**E**) The effect of NBAT1 knockdown on AGS cells. (**F**) The effect of NBAT1 overexpression on BGC-823 cells. (**G**) The apoptosis of AGS cells expressing control and NBAT1 shRNAs was measured by flow cytometry. (**H**) The apoptosis of control and NBAT1 overexpressed BGC cells expressing control and NBAT1 shRNAs was measured by flow cytometry. Data are shown as mean ± S.D.; *P<0.05.

### NBAT1 suppresses GC migration and invasion

To examine the effect of NBAT1 on cell migration and invasion capacity, transwell assays were performed. As shown in Figure 3A, deletion of NBAT1 promoted migration and invasion in AGS cells. In contrast, migratory and invasive capacity of BGC-823 cells was significantly repressed by NBAT1 overexpression (Figure 3B). These findings revealed that NBAT1 potentially influenced the GC progression through affecting cell migration and invasion.

**Figure 3:** NBAT1 suppresses GC migration and invasion (**A**,**B**) The migration and invasion of GC cells with NBAT1 alteration was detected by Transwell assay. Data are shown as mean ± S.D.; *P<0.05.

### NBAT1 inhibits proliferation, migration, and capillary tube formation of HUVECs

To ascertain the effects of NBAT1 on tumor angiogenesis, we employed tube formation by HUVECs for further investigation. As HUVECs can spontaneously form 3D tubular capillary-like network in Matrigel culture, which is a well-established cell model to study angiogenesis. We compared the functional effects of HUVECs using culture medium from control and NBAT1-overexpressing BGC-823 cells. After treatment of medium from BGC-823 cells with NBAT1 overexpression, HUVECs exhibited decreased cell proliferation (Figure 4A) and migration (Figure 4B), and formed less capillary tubes than control cells (Figure 4C). Conversely, the culture medium from AGS cells with NBAT1 knockdown significantly facilitated proliferation and migration of HUVECs (Figure 4D,E), and formed more capillary tubes relative to control cells (Figure 4F). These results indicate that NBAT1 represses the angiogenesis during GC progression.

**Figure 4:** NBAT1 inhibits proliferation, migration, and capillary tube formation of HUVECs (**A**) Proliferation assays of HUVECs treated with conditioned medium from AGS cells with NBAT1 overexpression. (**B**) Transwell migration assay of HUVECs cultured with NBAT1-overexpressing AGS cell medium. (**C**) Matrigel capillary tube formation assay. HUVECs were seeded on to a plate precoated with Matrigel and incubated with conditioned medium from NBAT1-overexpressing AGS cells. (**D**) Proliferation assays of HUVECs treated with conditioned medium from BGC-823 cells with NBAT1 knockdown. (**E**) Transwell migration assay of HUVECs cultured with NBAT1 knockdown BGC-823 cell medium. (**F**) Matrigel capillary tube formation assay. HUVECs were seeded on to a plate precoated with Matrigel and incubated with conditioned medium from NBAT1 knockdown BGC-823 cells. Data are shown as mean ± S.D.; *P<0.05.

### NBAT1 induces degradation of Sox9

To investigate the mechanisms of NBAT1 in GC progression, we performed RNA pull-down and MS to identify the proteins which are associated with NBAT1. We found that transcriptional factor Sox9 was a potential NBAT1-interacting candidate. As we know, Sox9 plays critical roles to drive cancer development including proliferation, migration, invasion, and angiogenesis [13–15]. RIP assay was used to confirm the interaction of between NBAT1 and Sox9 (Figure 5A). The results showed that endogenous NBAT1 could be significantly enriched by anti-Sox9 antibody than nonspecific IgG. For further validation, we performed RNA pull-down assays using biotin-labeled NBAT1 and cellular extracts. As shown in Figure 5B, a strong signal was observed in proteins pulled down with NBAT1 RNA but not in samples bound with antisense NBAT1.

**Figure 5:** NBAT1 induces degradation of Sox9 (**A**) The RIP assay was performed to confirm the interaction between NBAT1 and Sox9. IgG was taken as negative control. (**B**) The RNA pull-down assay was performed to validate the interaction between NBAT1 and Sox9. S indicates sense NBAT1. AS indicates antisense NBAT1. AS was taken as the negative control. (**C**) The *Sox9* mRNA was not affected by NBAT1 overexpression. (**D**) The *Sox9* mRNA was not affected by NBAT1 knockdown. (**E**) The Sox9 protein level in GC cells with NBAT1 alteration was detected by Western blot. (**F**) Control and NBAT overexpressed BGC-823 cells were treated with cycloheximide (CHX) for indicated time points. The cell lysates were examined by Western blot using the indicated antibodies. A plot of normalized amount of Sox9 protein was shown. (**G**) Western blot of Sox9 expression in control and NBAT1 overexpressed cells treated with vehicle control or MG132. (**H**) Western blot of Sox9-associated ubiquitination in control and NBAT1 overexpressed cells treated with MG132. Data are shown as mean ± S.D.; *P<0.05.

We then explored the functional relationship between NBAT1 and Sox9. Neither knockdown nor overexpression of NBAT1 affected *Sox9* mRNA level (Figure 5C,D). Intriguingly, knockdown of NBAT1 up-regulated Sox9 protein level, while Sox9 expression was reduced by NBAT1 overexpression (Figure 5E), indicating that NBAT1 regulated the degradation of Sox9 protein. Moreover, AGS was treated with inhibitor of protein synthesis cycloheximide (CHX) to analyze the stabilities of Sox9 after NBAT1 overexpression. Up-regulation of NBAT1 dramatically shortened the half-life of Sox9 protein (Figure 5F). The decrease in Sox9 mediated NBAT1 overexpression was almost abolished by treatment of proteasome inhibitor MG132 (Figure 5G). Moreover, we observed that NBAT1 dramatically repressed ubiquitination level of Sox9 (Figure 5H). Together, these results suggested that NBAT1 interacts with Sox9 and induces its degradation.

### The tumor-suppressive function of NBAT1 is dependent on Sox9

Since NBAT1 plays a role in regulating Sox9 protein level, we performed rescue assays to validate whether Sox9 is involved in the NBAT1-mediated inhibition of malignant progression in GC cells. We restored the Sox9 expression in NBAT1 overexpressed BGC-823 cells (Figure 6A). Notably, Sox9 could reverse the decrease on proliferation, migration, and invasion of GC cells caused by NBAT1 overexpression (Figure 6B,C). Moreover, Sox9 rescued the HUVECs’ proliferation, migration, and tube formation suppressed by treatment of culture medium from NBAT1-overexpressing BGC-823 (Figure 6D,E).

**Figure 6:** The tumor-suppressive function of NBAT1 is dependent on Sox9 (**A**) Sox9 expression was restored in NBAT1 overexpressed BGC-823 cells. (**B**,**C**) Sox9 could reverse the decrease in proliferation (B), migration and invasion (C) of GC cells caused by NBAT1 overexpression. (**D**) Proliferation assay of HUVECs cultured in the condition medium of NBAT1 overexpressed BGC-823 cells with and without Sox9. (**E**) Transwell migration assay of HUVECs cultured in the condition medium of NBAT1 overexpressed BGC-823 cells with and without Sox9. (**F**) Matrigel capillary tube formation assay of HUVECs under the condition medium of NBAT1 overexpressed BGC-823 cells with and without Sox9. Data are shown as mean ± S.D.; *P<0.05.

### NBAT1 transcription is suppressed by Sox9

Finally, we investigated which transcript factor is involved in the down-regulation of NBAT1 in GC. We used the JASPAR CORE database to analyze the promoter of NBAT1. Interestingly, the results showed that Sox9 potentially binds to the NBAT1 promoter region (Supplementary Table S1). We then transfected AGS and BGC-823 cells with siRNAs especially targetting Sox9, and the result showed that NBAT1 expression was up-regulated after Sox9 silence (Figure 7A). Moreover, we designed three different primers that covered the Sox9-binding sites and used ChIP-qPCR assays to examine whether Sox9 could bind to these sites. As shown in Figure 7B, STAT3 could associate with NBAT1 promoter. We also constructed the luciferase reporter plasmids containing NBAT1 promoter region. Dual luciferase reporter assays demonstrated that deletion of Sox9 could increase the luciferase activity of NBAT1 promoter region (Figure 7C). These results indicate that NBAT1 is regulated by Sox9, and there is a negative feedback loop between Sox9 and lncRNA NBAT1.

**Figure 7:** Sox9 suppresses NBAT1 transcription (**A**) AGS and BGC-823 cells were transfected with siRNAs against Sox9. The Sox9 and NBAT1 expression was then detected by qRT-PCR. (**B**) ChIP-qPCR analysis of Sox9 occupancy in the NBAT1 promoter in GC cells. (**C**) Luciferase assays of the cells indicated that were transfected with pGL3-linc-UFC1 vector, the E2F1 vector, or an empty vector. (**D**) Schematic diagram of NBAT1 regulating malignant progression via association with Sox9 in GC. Data are shown as mean ± S.D.; *P<0.05.

## Discussion

Increasing evidence has reported that lncRNAs play a key role in the pathogenesis of diseases, and aberrant expression of lncRNAs are frequently observed in several cancers, including GC [16]. Here, we found that NBAT1 was significantly down-regulated in GC tissues and associated with tumor differentiation, tumor stage, and lymph node metastasis, suggesting a clinical pathological role of NBAT1 expression in GC patients. In addition, survival analysis demonstrated that GC patients with lower NBAT1 expression had a worse prognosis. These findings suggested that NBAT1 may act as a novel prognosis marker for GC patients.

To further explore the effect of NBAT1 on GC cell phenotypes, loss- and gain-of-function assays were performed. We observed that lncRNA NBAT1 overexpression significantly inhibited GC cell proliferation, migration, and invasion and promoted cell apoptosis, whereas NBAT1 knockdown exerted the opposite functions. Consistent with our findings, previous studies also demonstrated a suppressive activity of NBAT1 in proliferation, migration, and invasion of cancer cells [10,11,17]. Angiogenesis is considered as a critical step during cancer progression [18]. Our present study is the first one to show that HUVECs exhibited decreased proliferation and migration and formed less capillary tubes after treatment of medium from NBAT1-overexpressing GC cells.

SOX9 belongs to the family of SRY-related high-mobility-group box (SOX) transcription factors that regulates pluripotency, cell lineage differentiation, and tissue homeostasis [19]. Evidence reported that SOX9 regulates some of its target genes through regions of the genome containing large clusters of transcriptional enhancers [20]. Abnormal expression of Sox9 has been observed in some human cancers. Sox9 plays critical roles in cancer progression, which regulates serious genes transcription to promote cell proliferation, migration, invasion, and angiogenesis. For instance, Sox9 represses Claudin-8 expression to promote osteosarcoma cell proliferation [21]. Sox9 transcriptionally activates LASP-1 expression to increase cell proliferation, migration, and invasion in lung cancer [22]. Recent studies demonstrated that lncRNAs act as competitive endogenous RNA (ceRNA) to post-transcriptionally regulate Sox9 expression, such as SNHG14 and MALAT1 [23,24]. However, to date, whether lncRNAs are involved in the post-translational modification of Sox9 protein remains unclear. Here, RIP and RNA pull-down assays demonstrated a direct interaction between NBAT1 and Sox9. In addition, overexpression of NBAT1 reduced Sox9 protein level and increased its ubiquitination level, indicating that NBAT1 is important for the stability of Sox9 protein. However, the exact mechanism by which NBAT1 induces Sox9 degradation needs further exploration. We speculated that NBAT1 may recruit some E3 ubiquitin ligase to promote Sox9 degradation. A recent study also demonstrated a similar regulation between lncRNA and its interacting protein. lnc-UICC directly interacted with the p-STAT3, and increased its protein stability. Moreover, STAT3 could bind to the lnc-UICC promoter to enhance its transcription, suggesting that there exists a positive feedback loop between lnc-UICC and STAT3 [25].

Of note, one of the most interesting findings from the present study is that Sox9 can also regulate expression of NBAT1. We analyzed the mechanism of NBAT1 down-regulation in GC. Intriguingly, we found that Sox9 could directly bind to NBAT1 promoter region and inactivate its transcription, suggesting that there exists a negative feedback loop between Sox9 and NBAT1. Other studies have also reported similar regulating mechanisms. For example, lncRNA HCP5 increases RUNX1 expression in glioma cells, while overexpression of RUNX1 can up-regulate HCP5 expression [26]. Our results further support the notion of a negative feedback regulating loop between lncRNAs and their interacting proteins, and suggest that this loop might be critical during GC initiation and development.

In conclusion, our current study highlights the importance of association between NBAT1 and Sox9 in regulation of GC progression. Down-regulation of NBAT1 could promote Sox9 expression, thereby promoting a series of oncogenic functions in GC cells. Sox9 could then in turn silence NBAT1 expression, which forms a negative feedback loop (Figure 7D) and may provide a potential therapeutic strategy for GC treatment.

## Supporting information

**Supplemental Table 1:** Putative binding sites of in Sox9 NBAT1 promoter region

## Abbreviations

CCK-8: cell counting kit-8
GALNT5: Polypeptide N-Acetylgalactosaminyltransferase 5
GC: gastric cancer
HUVEC: human umbilical vein endothelial cell
HCP5: HLA Complex P5
HSP90: Heat shock protein 90
LASP-1: LIM and SH3 domain protein 1
lncRNA: long noncoding RNA
MALAT1: Metastasis Associated Lung Adenocarcinoma Transcript 1
NBAT: lncRNA neuroblastoma associated transcript 1
qRT-PCR: quantitative real-time PCR
RIP: RNA immunoprecipitation
RUNX1: Runt-related transcription factor 1
SNHG14: Small Nucleolar RNA Host Gene 14
SOX: SRY-related high-mobility-group box
STAT3: Signal transducer and activator of transcription 3
